This article has been retracted.

# BCNet: A Novel Network for Blood Cell Classification

**DOI:** 10.3389/fcell.2021.813996

**Published:** 2022-01-03

**Authors:** Ziquan Zhu, Siyuan Lu, Shui-Hua Wang, Juan Manuel Górriz, Yu-Dong Zhang

**Affiliations:** ^1^ School of Computing and Mathematical Sciences, University of Leicester, Leicester, United Kingdom; ^2^ Department of Signal Theory, Networking and Communications, University of Granada, Granada, Spain; ^3^ Guangxi Key Laboratory of Trusted Software, Guilin University of Electronic Technology, Guilin, China

**Keywords:** blood cells, convolutional neural network, randomized neural network, ResNet-18, transfer learning

## Abstract

**Aims:** Most blood diseases, such as chronic anemia, leukemia (commonly known as blood cancer), and hematopoietic dysfunction, are caused by environmental pollution, substandard decoration materials, radiation exposure, and long-term use certain drugs. Thus, it is imperative to classify the blood cell images. Most cell classification is based on the manual feature, machine learning classifier or the deep convolution network neural model. However, manual feature extraction is a very tedious process, and the results are usually unsatisfactory. On the other hand, the deep convolution neural network is usually composed of massive layers, and each layer has many parameters. Therefore, each deep convolution neural network needs a lot of time to get the results. Another problem is that medical data sets are relatively small, which may lead to overfitting problems.

**Methods:** To address these problems, we propose seven models for the automatic classification of blood cells: BCARENet, BCR5RENet, BCMV2RENet, BCRRNet, BCRENet, BCRSNet, and BCNet. The BCNet model is the best model among the seven proposed models. The backbone model in our method is selected as the ResNet-18, which is pre-trained on the ImageNet set. To improve the performance of the proposed model, we replace the last four layers of the trained transferred ResNet-18 model with the three randomized neural networks (RNNs), which are RVFL, ELM, and SNN. The final outputs of our BCNet are generated by the ensemble of the predictions from the three randomized neural networks by the majority voting. We use four multi-classification indexes for the evaluation of our model.

**Results:** The accuracy, average precision, average F1-score, and average recall are 96.78, 97.07, 96.78, and 96.77%, respectively.

**Conclusion:** We offer the comparison of our model with state-of-the-art methods. The results of the proposed BCNet model are much better than other state-of-the-art methods.

## Introduction

Blood cells can spread throughout the body by the blood. There are three types of blood cells in mammals: 1) Red blood cells: transporting oxygen is the main function. 2) Leukocytes: mainly play the role of immunity when the body is invaded by bacteria. At that time, leukocytes can focus on the invasion site of bacteria, surround the bacteria, and swallow them. 3) Platelets: which are very important in hemostasis.

Most blood diseases, such as chronic anemia, leukemia (commonly known as blood cancer), and hematopoietic dysfunction, are caused by environmental pollution, substandard decoration materials, radiation exposure, and long-term use of certain drugs. They are all insidious, and the early symptoms are very mild and easy to ignore. Therefore, it is necessary to detect the number of various blood cells regularly. After increasing menstruation and skin purpura, detecting blood cells in time is necessary. By detecting the various blood cells in the blood, it can help doctors diagnose these diseases. Thus, it is vital to classify the blood cell images. In this paper, we automatically classify three cell types that affect neonatal blood cells. This blood cell image data are from the blood cell data set published on the Kaggle website (Mooney, 2017). However, Some diseases and their complications have no significant effect on neutrophil dynamics (Manroe et al., 1979). Therefore, it will not be tested in this paper. In a blood examination of the patient, medical professionals create a slide coated with blood, fix the slide, stain with chemical reagents such as Wright Gimsa and hematoxylin-eosin, and then carefully observe the blood cell changes (Ryu et al., 2020). It takes a long time for doctors to complete a blood cell test. However, the test results are also easily affected by the dyeing quality.

Researchers and practitioners try to classify blood cells based on computer technology. Salau and Jain (2021) proposed a method to predict Akt protein cells based on ML technology of multilayer perceptron (MLP) and radial basis function (RBF). Finally, the accuracy of this paper was 99.93%. Dudaie et al. (2020) put forward a model, based on a digital holographic microscope and machine learning, to detect and classify untouched cancer cells. In the experiment, the throughput was 15 cells per second. According to the experimental process’s cell flow morphology and quantitative phase characteristics, the accuracy can reach 92.56%. Marostica et al. (2021) suggested using a deep convolutional neural network for the detection and diagnosis of renal cancer. This method linked the quantitative pathological model with the patient’s genome map and prognosis. Finally, the AUC value of malignant tumors in the detection and validation cohort was 0.964–0.985. Wagner and Yanai (2018) developed a hierarchical machine learning framework called Moana. Moreover, the framework could construct a classifier in heterogeneous scRNA-Seq data sets. Begambre et al. (2021) proposed a low-cost classification approach by using artificial intelligence and computer vision to detect leukocytes. The final accuracy was 96.4%. Liang et al. (2018) introduced a recurrent neural network framework (CNN – RNN) that combined CNN and RNN. The framework can help to understand the image content and learn its characteristics. They tested and compared with other CNN models, and finally, they concluded that their proposed network model can better complete blood cell classification. Bur et al. (2019) presented an automatical system for detecting occult lymph node metastasis in clinical lymph node-negative oral squamous cell carcinoma (OCSCC). They finally got an AUC value of 0.840. Kocak et al. (2018) proposed to use texture analysis for the classification of renal cell computed tomography (CT) texture analysis. Zhang et al. (2017) employed a CNN to classify cervical cells. Finally, the accuracy of the method is 98.3%, and the area under the curve is 0.99. Şengür et al. (2019) presented a system that was a combination of machine learning (ML) with graphics processing (IP) to measure and classify leukocytes. The accuracy of the depth feature was 82.9%, the shape feature was 80.0%, and the accuracy of combining the two was 85.7%. Özel Duygan et al. (2020) expanded and accelerated microbiota analysis by a supervised algorithm. Imran Razzak and Naz (2017) proposed an effective contour-aware segmentation method. The method was based on a fully traditional network structure. In the classification process, they used extreme machine learning to extract CNN features from each unit. Habibzadeh et al. (2018) proposed a preprocessing algorithm for color distortion, bounding box distortion, and image flip mirror. Then, they used Inception and ResNet architecture to extract and recognize the characteristics of leukocytes. They obtained an accuracy of 98.33% and an AUC value of 0.9833. Lei et al. (2018) presented a classification framework for cell images to handle the challenges of intragroup changes caused by uneven illumination. The framework was based on the deeply supervised residual network. Kihm et al. (2018) presented a CNN based on machine learning to automatically classify the morphology of red blood cells in blood flow. Khamparia et al. (2020) presented an artificial intelligence system that was driven by the internet of healthy things for the detection of cervical cancer. Experiments show that the ResNet50 training model got the highest accuracy of 97.89%. Varghese (2020) classified four types of blood cells by using machine learning. Kan (2017) modeled the segmentation and tracking of individual cells and the reconstruction of phylogenetic trees using ML in optical microscope experimental image analysis. Wedin and Bengtsson (2021) used three classifiers to classify the cell types of mouse digital reconstruction images. The three classifiers were CNN, random forest classifier, and support vector classifier. Feng et al. (2018) proposed a method combining supervised machine learning and diffraction images to detect and classify different stages of apoptosis. Finally, the accuracy of this method was more than 90%. Su et al. (2020) suggested generating lighting patterns in the cells by single-mode fiber cytometry. Iliyasu and Fatichah (2017) proposed a new method (Qfuzzy) to extract and classify cervical smear cells’ characteristics based on particle swarm optimization and k-nearest neighbors. Alom et al. (2018) presented a new system to classify and detect colon cancer. This method combined the densely connected convolutional network (DCRN) and the recurrent residual u Network (R2U-Net).

It can be concluded from the above latest research analysis that most of the cell classification is based on the manual feature, machine learning classifier or the deep convolution neural network model (Jiao et al., 2019a). However, manual feature extraction is a very tedious process, and the results are usually unsatisfactory. Manually labeling the complete set to only consider the real information in that image is an unaffordable task. On the other hand, the deep convolution neural network is usually composed of massive layers, and each layer has many parameters (Jiao et al., 2019b). Therefore, each deep convolution neural network needs a lot of time to get the results. Another problem is that medical data sets are relatively small, which may lead to overfitting problems.

To deal with these problems described above, we propose seven models for the automatic classification of blood cells. The contributions of this paper are summarized as below:

- Seven models are proposed to automatically classify blood cells: BCARENet, BCR5RENet, BCMV2RENet, BCRRNet, BCRENet, BCRSNet, and BCNet.
- The BCNet model is the best model among the four proposed ensemble models after statistical experiments.
- After comparison, the proposed BCNet is better than the other three individual models.
- Three RNNs are selected to substitute the last four layers of the trained transferred ResNet-18 to shorten training time.
- The outputs of the BCNet are generated based on predictions from three RNNs using the majority voting.

In the proposed BCNet model, there are three randomized neural networks (RNNs), and all of them are feedforward neural networks with a single hidden layer. They are random vector functional link (RVFL), Schmidt neural network (SNN), and extreme learning machine (ELM). The number of parameters required in randomized neural networks (RNNs) is far less than that required by the deep convolution neural network model. Therefore, the proposed BCNet structure can avoid the problems of overfitting and greatly shorten training time and cycle.

The framework of this paper is as follows. *Material* section introduces the used materials in this paper. *Methodology* section presents the details and explanation of the proposed BCNet. The experiment settings and results of the BCNet are included in *Experiment Settings and Results* section. *Conclusion* section is about the conclusion.

## Material

This blood cell image data can be downloaded on the Kaggle website (Mooney, 2017). However, Some diseases and their complications have no significant effect on neutrophil dynamics (Manroe et al., 1979). And therefore, it will not be tested in this paper. We selected three cell types for training and testing. The three cell types are eosinophils, lymphocytes, and monocytes, as shown in Supplementary Figure S1A.

Eosinophils are a component of leukocytes. It is a hematopoietic stem cell-derived from bone marrow. Parasites and bacteria are eliminated by the Eosinophils. The lymphocyte is the smallest white blood cell which is produced by the Lymphatic organs. It is one of the most important components of the body’s immune. Monocytes are the largest blood cells in the blood, which are the irreplaceable component of the human defense system.

There are about 3,000 images Table 1 for each of three different cell types: Eosinophil, Lymphocyte, and Monocyte, respectively. The information of the data set is given in Supplementary Figure S1A. For training our models in this study, we encode the labels as: ${\left[100\right]}^{T}$ , ${\left[010\right]}^{T}$ , and ${\left[001\right]}^{T}$ , which represents Eosinophil, Lymphocyte, and Monocyte, respectively.

## Methodology

At present, many diagnostic systems based on artificial intelligence are used to analyze and classify images (Sheng et al., 2021; Jiao et al., 2021a). It is inevitable to extract the features of images for analyzing and classifying images (Jiao et al., 2021b). However, because each image contains a lot of information, extracting the discrimination rate features is difficult. With the continuous progress of computer vision technology and machine learning, many models have achieved great success, such as convolution neural networks (CNN) (Jiao et al., 2020a). The convolution layer in the CNN model can significantly reduce the parameters to reduce the computation, as shown in Figure 1A. The pooling layer further reduces the dimension of features while maintaining the dominant information (Jiao et al., 2018), as shown in Figure 1B.

**FIGURE 1:** Explanations of CNN. **(A)** Convolution layer flow chart. **(B)** An example of average and max pooling. **(C)** Activation function.

### Proposed BCNet

With more and more research on CNN, there are many CNN models (Jiao et al., 2019c), such as DenseNet (Huang et al., 2017), VGG (Simonyan and Zisserman, 2014), MobileNet (Sandler et al., 2018), EfficientNet (Tan and Efficientnet, 2019), AlexNet (Krizhevsky et al., 2017), ResNet (He et al., 2016), SqueezeNet (Iandola et al., 2016), and so on. This paper proposes seven models for the automatic classification of blood cells: BCARENet, BCR5RENet, BCMV2RENet, BCRRNet, BCRENet, BCRSNet, and BCNet. The BCNet model is the best model among the seven proposed models. The flowchart of our model is given in Figure 2A. The pseudocode of our model is shown in Table 2. The backbone model in our method is selected as the ResNet-18, which is pre-trained on the ImageNet set. We transfer the ResNet-18 model. After that, the transferred ResNet-18 is trained on the processed training set. Compared with ResNet-18, the training time of randomized neural networks is much shorter. To improve the performance of the proposed model, the end four layers of the trained transferred ResNet-18 model are replaced by three randomized neural networks (RNNs) which are RVFL, ELM, and SNN. The features *F* extracted from FC256 layer are used to train RVFL, ELM, and SNN. Because the randomized neural network parameters from the input layer to the hidden layer are random, we use the ensemble of the predictions of the three RNNs to improve the robustness of the network. The final outputs of our BCNet are generated by the ensemble of the predictions from the three randomized neural networks by the majority voting. To better verify the performance of our proposed BCNet model, we use multi-classification indexes to evaluate it.

**FIGURE 2:** Explanation of the proposed BCNet. **(A)** The flowchart of the proposed BCNet. **(B)** Original block. **(C)** Residual learning. **(D)** The transfer learning in the ResNet-18.

**TABLE 1:** The details of the data set.

	Eosinophil	Lymphocyte	Monocyte
Training set	2,497	2,483	2,478
Testing set	623	620	620

**TABLE 2:** Pseudocode of the proposed BCNet.

Step 1: Load the pre-trained ResNet-18.
Step 2: Divide the blood cell data set into training and testing sets.
Step 3: Preprocessing
Resize samples in the training and testing set based on the input size of ResNet-18.
Step 4: Generate the transferred ResNet-18.
Step 4.1: Remove FC1000, softmax, and classification layer from the pre-trained ResNet-18.
Step 4.2: Add FC256, ReLU, FC3, softmax, and classification layer.
Step 5: Train the transferred ResNet-18.
Step 5.1: Input is the processed training set.
Step 5.2: Target is the corresponding labels.
Step 6: Replace the last 4 layers of the trained transferred ResNet-18 with three RNNs.
Step 7: Extract features *F* as the output of the FC256 layer.
Step 8: Train the three RNNs on the extracted features *F* and the labels.
Step 8.1: Input is the extracted features *F*.
Step 8.2: Target is the labels of the processed training set.
Step 9: Add the majority voting layer.
Step 9.1: Ensemble the predictions of the three RNNs.
Step 9.2: Majority voting of the ensemble of the predictions from the three RNNs.
Step 9.3: The whole network is named BCNet.
Step 10: Test the trained BCNet on the processed testing set.
Step 11: Report the classification performance of the trained BCNet.

### Backbone of Proposed BCNet

The activation function (Jiao et al., 2020b) is added to activate some neurons in the CNN model, and the activated neurons are transmitted to the next layer, as shown in Figure 1C. If the activation function is not added, the neurons of each layer of CNN are linear.

However, when the neurons of each layer are nonlinear, it is challenging to implement identity mapping (He et al., 2016) in the training iteration. If the number of layers is deepened for a trained network structure, it is not simply stacking more layers but stacking one layer to make the output after stacking the same as before stacking and then continuing training. In this case, it is reasonable that the training results should not be worse because the level before adding layers has been taken as the initial before the training starts. However, the experimental results show that the results will be worse after the network layers reach a certain depth, which is the problem of degradation. This shows that the traditional nonlinear expression of multilayer network structure is difficult to represent identity mapping, as shown in Figure 2B. In this paper, we use the residual mechanism to deal with this problem. A stacked-layer structure is shown in Figure 2C.

When the input is *X*, the original learned feature is recorded as *T*(*X*), and *L*(*X*) is obtained through the residual network formula, which is as follows:

L(X)=T(X)−X (1)

Through the above formula conversion, the original learned feature is:

T(X)=L(X)+X (2)

Compared with direct learning, residual learning is a better method for original features. Because when the residual is 0, the residual learning can at least carry out the identity mapping. Thus, it would not have any bad influences on the system performance. When the residual is not 0, it can learn new features from other layers.

The backbone model in our method is selected as the ResNet-18, which is pre-trained on the ImageNet set. We transfer the ResNet-18 model. The transfer learning in the ResNet-18 is shown in Figure 2D. We replace FC1000 with FC3 because there are three types of images of blood cells in this paper and add FC256 to reduce dimensional differences. In addition, we delete the last four layers of the trained transferred ResNet-18 model and add three RNNs. Therefore, the trained transferred ResNet-18 model is the proposed BCNet feature extractor in this paper. FC256 is the feature layer.

### RNNs Ensemble in BCNet

With the continuous research of the CNN models, the CNN models are becoming more and more excellent (Ji et al., 2021). Especially for training and testing on large data sets, the CNN models achieve better and better results. In the proposed BCNet model, the end four layers of the trained transferred ResNet-18 are replaced by three randomized neural networks (RNNs). The three RNNs are RVFL (Pao et al., 1994), ELM (Huang et al., 2006), and SNN (Schmidt et al., 1992).

As shown in Figure 3, these three diagrams are 1) RVFL, 2) ELM, and 3) SNN, respectively. The blue box represents the input, the hidden nodes in the hidden layer are shown by the orange circle, and the pink box is the output. It can be seen from Figure 3 that the main difference between SNN and ELM is that there are biases in the SNN. The main difference between RVFL and the other two RNNs (SNN and ELM) is that they can be connected directly from the input layer to the output layer in RVFL.

**FIGURE 3:** Structure of three RNNs. **(A)** RVFL. **(B)** ELM. **(C)** SNN.

Although the structures of the three RNNs are more and less different, the calculation steps of the three RNNs are similar. First, for *N* arbitrary distinct samples, set a data set with the *i*-th sample as $\left(x_{i},y_{i}\right)$ :

$$x_{i}={\left(x_{i1},\ldots ,x_{in}\right)}^{T}\in R^{n},\;i=1,\ldots ,N,$$ (3)

$$y_{i}={\left(Q_{i1},\ldots ,\;Q_{im}\right)}^{\text{T}}\in {\text{R}}^{m},\;i=1,\ldots ,\;N,$$ (4)

where *n* represents the input dimension, *m* represents the output dimension.

The calculation of three RNNs: $A_{j}$ is the weight vector connecting the *j*-th hidden node and the input nodes, $K_{j}$ is the bias of the *j-*th hidden node. Thus, the output matrix of the hidden layer containing *Z* hidden nodes can be calculated:

$$U_{\mathrm{RVFL}\left(i\right)}=\text{concat}\left(X,V\right),$$ (5)

where $X={\left(x_{1},\ldots ,x_{N}\right)}^{T}$ is the input characteristic matrix. **V** is the random hidden mappings. The formula is as follows:

$$V_{\mathrm{RVFL}\left(i\right)}=\sum_{j=1}^{Z}g\left(A_{j}x_{i}+K_{j}\right),\;i=1,\ldots ,N,$$ (6)

where *g*() represents the sigmoid function.

For ELM, the equation is as follows:

$$U_{\mathrm{ELM}\left(i\right)}=\sum_{j=1}^{Z}g\left(A_{j}x_{i}+K_{j}\right),\;i=1,\ldots ,N.$$ (7)

For SNN, the formula is as follows:

$$U_{\mathrm{SNN}\left(i\right)}=\sum_{j=1}^{Z}g\left(A_{j}x_{i}+K_{j}\right),\;i=1,\ldots ,N.$$ (8)

The final output weights (**W**) are obtained by pseudo-inverse:

$$W=U_{\mathrm{net}}^{+}Y,\;\text{net}=\text{ELM}\;\text{or}\;\text{RVFL},$$ (9)

where $U_{\mathrm{net}}^{+}$ denotes the pseudo-inverse matrix of $U_{\mathrm{net}}$ and $Y={\left(y_{1},\ldots ,y_{N}\right)}^{T}$ is the ground-truth label matrix of the dataset.

Because SNN adds biases (**E**) on the output layer, its formula is:

$$\left(W,E\right)=U_{\mathrm{net}}^{+}Q,$$ (10)

where $U_{\mathrm{net}}^{+}$ denotes the pseudo-inverse matrix of $\left(\begin{array}{c} U_{\mathrm{net}}\\ 1 \end{array}\right)$ .

For improving the robustness of BCNet, the final outputs of our model are generated by the ensemble of the predictions from the three randomized neural networks by the majority voting. Suppose given an image $s_{am}$ , and $L\left(s_{am}\right)$ is the function of the final output, $Q_{\alpha }$ , $Q_{\beta }$ , and $Q_{\gamma }$ mean three predictions from three RNNs for image $s_{am}$ , respectively.

$$L\left(s_{am}\right)=\{\begin{array}{cc} Q_{t},\;if\;\exists Q_{t}==Q_{b},\; & t,b\in \left\{\alpha ,\beta ,\;\gamma \right\}\\ {\left[100\right]}^{T}, & \text{otherwise} \end{array},$$ (11)

where ${\left[100\right]}^{T}$ denotes the Eosinophil.

### Other Proposed Models

Compared with ResNet-18, the training time of randomized neural networks is much shorter. We replace the end four layers of the trained transferred ResNet-18 model with three RNNs: RVFL, ELM, and SNN, respectively, and three models are obtained: BCRRNet, BCRENet, and BCRSNet. The details of the proposed three individual models are given in Table 3.

**TABLE 3:** Other proposed models.

Proposed individual model (Abbreviation)	Meaning	Training
ResNet-18-RVFL (BCRRNet)	We select RVFL to substitute the end four layers of the trained transferred ResNet-18 and get BCRRNet.	RVFL in the BCRRNet is trained by the features which are extracted from FC256.
ResNet-18-ELM (BCRENet)	We select ELM to substitute the end four layers of the trained transferred ResNet-18 and get BCRENet.	ELM in the BCRENet is trained by the features which are extracted from FC256.
ResNet-18-SNN (BCRSNet)	We select SNN to substitute the end four layers of the trained transferred ResNet-18 and get BCRSNet.	SNN in the BCRSNet is trained by the features which are extracted from FC256.
Proposed ensemble model (Abbreviation)	Meaning	Training
AlexNet-RNNs-En (BCARENet)	The pre-trained AlexNet is the backbone of the BCARENet and the results of the BCARENet are generated by the ensemble of the predictions from the three RNNs by the majority voting.	The trained transferred AlexNet is obtained by training the transferred AlexNet on the processed training blood cell data set. Then, three RNNs in the BCARENet are trained by the features which are extracted from FC256.
ResNet-50-RNNs-En (BCR5RENet)	The pre-trained ResNet-50 is the backbone of the BCR5RENet and the results of the BCR5RENet are generated by the ensemble of the predictions from the three RNNs by the majority voting.	The trained transferred ResNet-50 is obtained by training the pre-trained ResNet-50 on the processed training blood cell data set. Then, three RNNs in the BCR5RENet are trained by the features which are extracted from FC256.
MobileNet-V2-RNNs-En (BCMV2RENet)	The pre-trained MobileNet-V2 is the backbone of the BCMV2RENet and the results of the BCMV2RENet are generated by the ensemble of the predictions from the three RNNs by the majority voting.	The trained transferred MobileNet-V2 is obtained by training the pre-trained MobileNet-V2 on the processed training blood cell data set. Then, three RNNs in the BCMV2RENet are trained by the features which are extracted from FC256.

Because the randomized neural network parameters from the input layer to the hidden layer are random, we use the ensemble of the outputs of the three RNNs to improve the robustness of the network. This paper’s other three proposed ensemble models are BCARENet, BCR5RENet, and BCMV2RENet, respectively, as shown in Table 3. These three proposed ensemble models select the pre-trained AlexNet, the pre-trained ResNet-50, and the pre-trained MobileNet-V2 as their backbones. Three backbones are trained as the operations to get the trained transferred ResNet-18.

### Evaluation

We use multi-classification indexes to evaluate the proposed BCNet. In this paper, there are three categories (c=1,…,3) . When the label of one category is set to positive, the labels of the other two categories are set to negative. When the label of the B category is positive, the definitions of true positive (TP), true negative (TN), false negative (FN), and false positive (FP) are shown in Supplementary Figure S1B.

Four multi-classification indexes are applied to this paper. They are accuracy, average recall, average F1-score, and average precision. The formulas of the three indexes (precision, recall, and F1) pre category are as follows:

$$\{\begin{array}{l} \text{precision}\left(c\right)=\frac{\text{TP}\left(c\right)}{\text{TP}\left(c\right)+\text{FP}\left(c\right)}\\ \text{recall}\left(c\right)=\frac{\text{TP}\left(c\right)}{\text{TP}\left(c\right)+\text{FN}\left(c\right)}\\ \text{F}1\left(c\right)=\frac{2\times \text{prcision}\left(c\right)\times \text{recall}\left(c\right)}{\text{precision}\left(c\right)+\text{recall}\left(c\right)} \end{array},c=1,\ldots ,3.$$ (12)

In this paper, we use the macro average for multi-classification indexes calculation. The formulas for calculating the three multi-classification indexes (average-precision, average-recall, and average-F1) are below:

$$\{\begin{array}{l} \text{average}-\text{precision}=\frac{\sum_{c=1}^{3}\text{precision}\left(c\right)}{3}\\ \text{average}-\text{recall}=\frac{\sum_{c=1}^{3}\text{recall}\left(c\right)}{3}\\ \text{average}-\text{F}1=\frac{\sum_{c=1}^{3}\text{F}1\left(c\right)}{3} \end{array}$$ (13)

The accuracy in multi-classification is the proportion of correctly classified samples in total samples.

## Experiment Settings and Results

### Experiment Settings

We adjust the parameters of the proposed BCNet model in this paper. Our mini-batch size for each time is 50. To avoid the overfitting problems, we set the max-epoch to 2. Based on experience, we set the learning rate to 1e-4. We set a super parameter in the three RNNs. The number of hidden nodes Z is 400, which is determined based on the input dimension of RNNs. The hyper-parameter settings of BCNet are demonstrated in Supplementary Figure S1C.

### The Performance of BCNet

The blood cell data set has been divided into the experiment’s training and testing set. Table 4 shows the test confusion matrix.

**TABLE 4:** The test confusion matrix of BCNet.

		Predicted class		
		Eosinophil	Lymphocyte	Monocyte
Actual class	Eosinophil	623	0	0
	Lymphocyte	0	620	0
	Monocyte	60	0	560

The calculation principle of the four multi-classification evaluation indexes in this paper is shown in *Three Proposed Ensemble Models* section. There are three categories in this paper, and the results of each category are shown in Table 5.

**TABLE 5:** The results of each category.

Category	Precision (%)	Recall (%)	F1 (%)
Eosinophil	91.22	100	95.41
Lymphocyte	100	100	100
Monocyte	100	90.32	94.92

The specific calculations of four multi-classification indexes are:

$$\{\begin{array}{l} \text{accuracy}=\frac{\left(623+620+560\right)}{\left(623+620+560+60\right)}=96.78\%\\ \text{average}-\text{precision}=\frac{91.22\%+100\%+100\%}{3}=97.07\%\\ \text{average}-\text{recall}=\frac{100\%+100\%+90.32\%}{3}=96.77\%\\ \text{average}-\text{F}1=\frac{95.41\%+100\%+94.92\%}{3}=96.78\% \end{array}$$ (14)

### Comparison of the Proposed BCNet With Other Proposed Models

The confusion matrixes of other proposed models are shown in Table 6. The comparison of the proposed BCNet with the other proposed models is shown in Table 7. For a more intuitive view, the comparison of the proposed BCNet with the other proposed models is shown in Figure 4. As shown in the table and figure, we can conclude that the proposed BCNet has better performance than the other proposed models.

**TABLE 6:** Confusion matrixes of other proposed models.

	Predicted				
			Eosinophil	Lymphocyte	Monocyte
BCRRNet (Individual)	Actual	Eosinophil	621	2	0
		Lymphocyte	0	619	1
		Monocyte	72	0	548
BCRENet (Individual)	**Predicted**				
			Eosinophil	Lymphocyte	Monocyte
	Actual	Eosinophil	623	0	0
		Lymphocyte	0	619	1
		Monocyte	68	0	552
BCRSNet (Individual)	**Predicted**				
			Eosinophil	Lymphocyte	Monocyte
	Actual	Eosinophil	623	0	0
		Lymphocyte	0	619	1
		Monocyte	65	0	555
BCARENet (Ensemble)	**Predicted**				
			Eosinophil	Lymphocyte	Monocyte
	Actual	Eosinophil	432	62	129
		Lymphocyte	7	600	13
		Monocyte	176	0	444
BCR5RENet (Ensemble)	**Predicted**				
			Eosinophil	Lymphocyte	Monocyte
	Actual	Eosinophil	550	73	0
		Lymphocyte	0	620	0
		Monocyte	90	0	530
BCMV2RENet (Ensemble)	**Predicted**				
			Eosinophil	Lymphocyte	Monocyte
	Actual	Eosinophil	582	35	6
		Lymphocyte	8	601	11
		Monocyte	153	7	460

**TABLE 7:** Comparison of the proposed BCNet with other proposed models.

Model	Accuracy (%)	Average-precision (%)	Average-recall (%)	Average-F1 (%)
BCRRNet (Individual)	95.97	96.37	95.97	96.17
BCRENet (Individual)	96.30	96.66	96.29	96.47
BCRSNet (Individual)	96.46	96.79	96.45	96.62
BCARENet (Ensemble)	79.23	78.88	79.24	79.01
BCR5RENet (Ensemble)	91.25	91.80	91.26	91.24
BCMV2RENet (Ensemble)	88.19	89.41	88.18	88.08
**BCNet (Ours)**	**96.78**	**97.07**	**96.77**	**96.78**

**FIGURE 4:** Comparison of the proposed BCNet with other proposed models.

### Explainability of the Proposed BCNet

In this section, we explain the proposed BCNet model. Usually, it’s hard to understand how deep models make predictions. However, with the help of Gradient-weighted class activation mapping (Grad-CAM) (Selvaraju et al., 2017), we can observe where the deep model pays attention. The Gradient-weighted class activation mapping is shown in Figure 5. In the raw image, eosinophilic nuclei are mostly C-type, S-type, or irregular type. Lymphocyte nuclei are quasi round or round, often on one side. The nuclei of monocytes are irregular, distorted, and overlapped. As can be seen from the heatmap, there are probably three red, blue, and orange colors on the Grad-CAM figure. The red area represents the place with the closest attention, the orange area is close attention, and the blue area has the lowest attention.

**FIGURE 5:** Explainability of our proposed BCNet. **(A)** One raw image of Eosinophils. **(B)** One raw image of Lymphocytes. **(C)** One raw image of Monocytes. **(D)** Heatmap of **(A)**. **(E)** Heatmap of **(B)**. **(F)** Heatmap of **(C)**.

### Comparison With Other State-Of-The-Art Methods

To better show the superiority of the proposed BCNet in this paper, we compare it with other state-of-the-art methods. These state-of-the-art methods are CNN+RNN (Liang et al., 2018), ML (Kihm et al., 2018), Q-fuzzy (Iliyasu and Fatichah, 2017), and DCRN+R2U (Alom et al., 2018). The comparison results are shown in Table 8. For a more intuitive view, the comparison chart is shown in Figure 6. It is not difficult to conclude from the figure and table that the experimental results of the proposed BCNet model are far better than these of other state-of-the-art methods.

**TABLE 8:** Comparison with other state-of-the-art methods.

Method	Accuracy	Average-precision	Average-recall	Average-F1	Source	Category
CNN+RNN Liang et al. (2018)	90.79%	—	—	—	Public	Four
ML Kihm et al. (2018)	86.70%	86.19%	86.25%	86.22%	Private	Three
Q-fuzzy Iliyasu and Fatichah (2017)	—	85%	86%	85%	Public	Seven
DCRN+R2U Alom et al. (2018)	91.14%	—	—	81.80%	Public	Four
BCNet (Ours)	96.78%	97.07%	96.77%	96.78%	Public	Three

**FIGURE 6:** Comparison with other state-of-the-art methods.

## Conclusion

The paper proposes seven models for the automatic classification of blood cells: BCARENet, BCR5RENet, BCMV2RENet, BCRRNet, BCRENet, BCRSNet, and BCNet. The BCNet model is the best model among the seven proposed models. The backbone model in our method is selected as the ResNet-18, which is pre-trained on the ImageNet set. To improve the performance of the proposed model, we replace the last four layers of the trained transferred ResNet-18 model with the three RNNs: RVFL, ELM, and SNN. The final outputs of our BCNet are generated by the ensemble of the predictions from the three randomized neural networks by the majority voting. We use four multi-classification indexes for the evaluation of our model. The accuracy, average precision, average F1-score, and average recall are 96.78, 97.07, 96.78, and 96.77%, respectively. We offer the comparison of our model with state-of-the-art methods. The results of the proposed BCNet model are much better than other state-of-the-art methods.

Although the proposed BCNet model in this paper has achieved excellent outputs, there are still some deficiencies. This paper mainly tests single cells but does not include overlapping cells and cell clusters tests. We do not detect all types of images in this data set. This paper uses only three types of this data set.

In future research, we will do more research about single cells, overlapping cells, and cell clusters classification and more methods to classify blood cells, such as CAD systems. At the same time, we will also use this method on other data sets.

## Data Availability

Publicly available datasets were analyzed in this study. This data can be found here: https://www.kaggle.com/paultimothymooney/blood-cells.
